The article "Classification of Electrocardiography Hybrid Convolutional Neural Network-Long Short Term Memory with Fully Connected Layer" was published in 2022. Journal: Comput Intell Neurosci.

# Classification of Electrocardiography Hybrid Convolutional Neural Network-Long Short Term Memory with Fully Connected Layer

**DOI:** 10.1155/2022/6348424

**Published:** 2022-07-11

**Authors:** Dhanagopal Ramachandran, R. Suresh Kumar, Ahmed Alkhayyat, Rami Q. Malik, Prasanna Srinivasan, G. Guga Priya, Amsalu Gosu Adigo

**Affiliations:** ^1^Centre for System Design, Chennai Institute of Technology, Chennai, Tamil Nadu, India; ^2^Department of Computer Technical Engineering, College of Technical Engineering, The Islamic University, Najaf, Iraq; ^3^Department of Medical Instrumentation Techniques Engineering, AI-Mustaqbal University College, Hillah 51001, Iraq; ^4^Department of Information Technology, R.M.D. Engineering College, Kaveripettai, Thiruvallur, Tamil Nadu, India; ^5^School of Electronics Engineering, Vellore Institute of Technology, Chennai, Tamil Nadu, India; ^6^Center of Excellence for Bioprocess and Biotechnology, Department of Chemical Engineering, College of Biological and Chemical Engineering, Addis Ababa Science and Technology University, Addis Ababa, Ethiopia

## Abstract

Electrocardiography (ECG) is a technique for observing and recording the electrical activity of the human heart. The usage of an ECG signal is common among clinical professionals in the collection of time data for the examination of any rhythmic conditions associated with a subject. The investigation was carried out in order to computerize the assignment by exhibiting the issue using encoder-decoder techniques, creating the information that was simply typical of it, and utilising misfortune appropriation to anticipate standard or anomalous information. On a broad variety of applications such as voice recognition and prediction, the long short-term memory (LSTM) fully connected layer (FCL) and the two convolutional neural networks (CNNs) have shown superior performance over deep learning networks (DLNs). DNNs are suitable for making high points for a more divisible region and CNNs are suitable for reducing recurrence types, LSTMs are appropriate for temporary displays, in the same way as CNNs are appropriate for reducing recurrence types. The CNN, LSTM, and DNN algorithms are acceptable for viewing. The complementarity of DNNs, CNNs, and LSTMs was investigated in this research by bringing them all together under the single architectural company. The researchers got the ECG data from the MIT-BIH arrhythmia database as a result of the investigation. Our results demonstrate that the approach proposed may expressively describe ECG series and identify abnormalities via scores that outperform existing supervised and unsupervised methods in both the short term and long term. The LSTM network and FCL additionally demonstrated that the unbalanced datasets associated with the ECG beat detection problem could be consistently resolved and that they were not susceptible to the accuracy of ECG signals. It is recommended that cardiologists employ the unique technique to aid them in performing reliable and impartial interpretation of ECG data in telemedicine settings.

The article "Classification of Electrocardiography Hybrid Convolutional Neural Network-Long Short Term Memory with Fully Connected Layer" was published in 2022. Journal: Comput Intell Neurosci.

## 1. Introduction

Electrocardiography (ECG) provides a significant amount of information about cardiovascular health and architecture, and it is the principal tool for diagnosing cardiac illness [1]. Arrhythmia is a highly frequent cardiac ailment that is well researched and understood by specialists in the field. Throughout the course of clinical practice, mistakes in diagnosis and inaccurate outcomes may occur due to the gap in expertise between experts and the absence of a smooth flow of information [2]. Programmable detection of arrhythmias and traceable confirmation of occurrences are critical because specialists should be assisted in distinguishing between arrhythmic events before they are seen.

For the most part, the diagnosis of arrhythmia has focused on screamed impulses from the electrocardiogram (ECG), manual extraction of components [3, 4], and pulse segmentation [5, 6]. Given the ambiguous complexity of the real scientific dataset, it is necessary to do thorough administration in order to mitigate the possible consequences of a diagnostic prediction inaccuracy. A full EKG signal, as illustrated in Figure 1, has been seen to include the QRS complex and P wave (current set in the electrocardiogram) and sometimes the T wave. Figure 1 shows the normal ECG, with ranges of the wave characteristics, as well as the wave features themselves. As a result, medical information technology has been widely employed to evaluate EHR data and accurately define the condition, based on artificial intelligence assessments combined with realistic methods. The following study has expanded group estimates to include algorithmic characterizations of blood pressure, such as K-nearest neighbor (KNN), Naive Bayes, and decision trees (DTs) [7]. In addition, three types of SVM classifications were developed with the goal of predicting cardiac pathology [8]. In order to identify cardiovascular conditions based on the SVM arrangement of heart sounds, it is advised that an automated classification system be used [9]. Recently, neural models have shown exceptional efficiency in terms of anticipating details and resolving a variety of structural challenges. Health care is increasingly relying on approaches of the deep learning in order to uncover new knowledge and control disease, particularly in the fields of diabetes, coronary artery disease, and cerebrum infection, using biomedical data [10]. There have been a few therapeutic implementations of deep learning, which can be seen more clearly in the [11] section. There are a number of useful neural system-based models that are mostly focused on correctly classifying cardiac diseases [12]. Scientists are currently experimenting with the use of convolutional neural networks (CNNs) to distinguish between various ECG signal classifications and to separate ECG information into normal versus pathological structures [13]. The RNN may also be used to detect probable infections by employing unambiguous EHR patient representations and presenting transitional linkages within EHR data events. Recently, researchers have used gated recurrent units (GRUs) and long short-term memory (LSTM) modules to predict cardiovascular disease risk and transient vascular infection [14]. As cutting-edge deep learning advances, convolutional computations will be employed to complete a number of extraction tasks. In contrast to morphology, the technique is less difficult and the signal efficiency criteria are less strict [15]. Researchers were able to recognize and characterize premature ventricular limits and ventricular ectopic beats using the one-dimensional convolutional neural network (1D CNN) developed by Li et al. [16]. It was claimed by [17] that comparable 1D CNN grouping may considerably increase system efficacy by arranging for more divisions of coronary artery problems than had ever been offered before. Some concerns in the literature on ECG arrhythmias remain unresolved, including the lack of ECG signal details during highlight mining or commotion cleaning, as well as a poor description of the internal mixture technique.

The article "Classification of Electrocardiography Hybrid Convolutional Neural Network-Long Short Term Memory with Fully Connected Layer" was published in 2022. Journal: Comput Intell Neurosci.

This work presents a 2D grayscale picture model that is entered into an LSTM together with deep 2D CNNs as a result of issues encountered. It is possible to avoid the loss of many ECG data points by converting the ECG to a 2D picture with a 1D signal, although this is more complicated. Due to the sensitive nature of the material, most current evaluations rely on restricted information. Preprocessing one-dimensional ECG data can have a significant impact on the absolute accuracy of one-dimensional ECG signals; therefore, most investigations would be cautious. More information and finer details can be obtained by converting 1D ECG data into 2D ECG images [18]. When converting data, is it required to separate each beat into its own distinct entity? Noise data may be overlooked by the convolution layer of the model, resulting in a false positive if all of the signals are separated. Automatic processes like filtering and feature extraction are not required for 2D ECG images. Assuming that noise data are almost certainly ignored by the pooling and convolution layers in these configurations, they preserve strategic separation from the question of how noise and precision are related in the process of producing a feature map. Photographs are also used as details in certain similar illness studies by numerous doctors [19, 20] instead of 1D signals to better grasp the ailment. 2D ECG images are more comparable to the path travelled by a cardiologist in the course of his or her research and identification of symptoms via visual perception when it comes to the detection and classification of rhythmic disturbances. In equipment such as ECG monitors, difficulties such as sluggish sampling rates and vibration would arise if an ECG signal was used that was only one dimension. ECG tracking robots will be able to use two-dimensional ECG images more regularly, which will help cardiac doctors diagnose arrhythmic illnesses. It is getting increasingly challenging to use the information development methods that have been used in previous studies because of the current properties of the 1D ECG data. Use the ECG signal to increase the planning data available, which will aid in the improvement of layout correctness. In order to support the CNN 2D methodology, which trained a single ECG image from several angles, we used a variety of alternative trimming approaches to enlarge the 2D ECG image. It is possible to use a 2D CNN to modularly highlight an automated ECG extraction, which would fix the current hand-planned waveform inclusions that are not robust enough for distinguishing tolerable variances in heartbeats. The recurrent neural network (RNN) can be used to learn from previous experiences as an alternate deep learning mechanism for LSTM to the 2D CNN design. All cells in the LSTM's input condition are conditional on the data's status and time components, which provides a strategic buffer against the problem of long-term dependence. In spite of the fact that data have been explicitly removed from the system, LSTM cells can retain and manage useful information [21]. Classification accuracy is greatly improved by combining LSTM and 2D CNN.

## 2. Related Work

Chest discomfort, suffering, and exhaustion, as well as an irregular heart rate and a slew of other symptoms, can all be traced back to cardiovascular disease. Heart disease can be diagnosed using a variety of factors. Age, gender, and other risk variables are taken into account. All of these risk factors, including alcohol intake, smoking, obesity, and a wide range of diseases such as asthma, are linked to each other in some way. There are a plethora of factors that make it challenging for doctors to accurately diagnose and assess heart illness. Traditional classification techniques such as support vector machines (SVMs), a priori algorithms, decision trees, and the hybrid random forest model [22, 23] have already been developed for classifying and analysing EHR data related to coronary disease expectancies. Using logistical recurrence and the Bayesian data definition, cardiovascular failure prediction has been proven and got an AUC score of 77% [24, 25]. Utilising logistic recurrence and a higher AUC score of 77%, this has been shown to be true using Bayesian data and the preferred methodology.

The article "Classification of Electrocardiography Hybrid Convolutional Neural Network-Long Short Term Memory with Fully Connected Layer" was published in 2022. Journal: Comput Intell Neurosci.

Convolutional neural networks (CNNs) and multilayer perceptrons (MLPs) were employed to review foetal pulse recordings with an 85% accuracy; a recurrent neural network (RNN) was also proposed in records with an 83% precision for the detection of abnormal heartbeat rhythms. Atrial fibrillation order was predicted using a long short-term memory organiser [26, 27], which achieved a 78% accuracy rate and a 79% F1 value in this job [28]. Computerized PCG signal analysis was also employed to identify the risk of programed auxiliary cardiac abnormalities (PACAs) in juvenile coronary heart disease diagnostics. To improve the accuracy of coronary disease applications, the BiLSTM estimate was taken into account when designing the bidirectional neural network architecture, which resulted in an increase in accuracy of 99.49% [29]. Biomedical researchers have a wide range of objectives when it comes to neural network performance, and the best results have been realised in clinical imaging using deep learning [30]. In order to improve automated clinical findings and suggest a strong morphological approach to real ECG chronicles, a generative adversarial network (GAN) was created. It has been used in conjunction with cardiovascular disease specialists who supported large absorptions of electronic clinical data by the LTSM model and ambulatory courses that were exposed by fictional substance with the BiLTSM [31, 32].

As new ideas like ensemble learning emerged to better the application of structures, established knowledge mining techniques saw their reach expand. In order to analyse and classify cardiac diseases based on their proximity and absence, the aim is to build a well-known ensemble learning model [33]. One can predict that the model's accuracy will be superior to that of top-tier findings. Instead of creating a single classification, the power of ensemble learning was utilised by completing predictions from a number of various classifiers, and AdaBoost computations and the bagging tree were used to lower the risk of heart disease in a case study [34]. A neural network-based ensemble strategy was proposed in order to produce a highly powerful classification approach and to offer a promising accuracy structure [35]. The example of ensemble learning model is hypothesised that LSTM-CNN-based identification of cardiovascular breakdown.

The article "Classification of Electrocardiography Hybrid Convolutional Neural Network-Long Short Term Memory with Fully Connected Layer" was published in 2022. Journal: Comput Intell Neurosci.

Training set mismatches can affect how existing arrangement models are displayed, and one of these elements is the presentation of existing arrangement models when they are used to show actual information. Predicted classifiers remain focused on a single class and have not summarised the information gathered during training. The approaches are edited nearest neighbors (ENNs), Smote, and Tomek [36] should be utilized during model construction to update the information for greater relevance [37]. Using an EKG-based heartbeat order ensemble learning system setup, the well-characterized presentation of a stable multiclass grouping issue was established [38].

## 3. Methodology

The MIT-BIH arrhythmias database was utilised to collect the study's data and observations, both of which can be accessed online. A total of 48 hours of data were collected from 48, 0.5-hour ECG signal reports from 47 different subjects using two conditions [7]. The R peak frequency of 360 hertz has been used to examine every single signal record. Unidentified cardiologists have offered their interpretations of these data in the form of anonymous comments. For the sake of data processing, electrocardiograms (ECGs) have been transformed into ECG images. Tests described in this research utilised lead II's specific symptoms as a guide: “V” for premature ventricular constriction (PVC), “L” for the left branch square block (LBSB), “N” for the standard signal rhythm (SSR), “A” for atrial premature beat (APB), “R” for the right bundle branch block (RBBB), “/” for paced beat (PAB), “E” for premature ventricular constriction (PVC), and “!” for ventricular fibrillation (VFW). Here, the nodal leanings were restricted to ventricular flutter and few beats that were not recognized as rhythms were built on that foundation. Most ECG arrhythmia investigations have failed to take into account the low criticality of these types of beats.  Figure 2 depicts the broad approaches.

### 3.1. Preprocessing

For each individual, the ECG signal lasts around 2–3 minutes on average. We separated the picture into tens of windows based on its growth. The morphology or range of the signal has no influence, and as a result, we do not clean or convert the signal in this case. Only the R-R signal [39] is isolated during the preprocessing stage. The approach adopted is incredibly required and effective even if the assumption of the signal is not made. In Figure 3, you can see that both signals have been upgraded to 188 with labels 1 and 0 for anomalous and unusual indications, respectively. A typical signal may have an average explanation; however, an abnormal signal may not have an explanation for such an extraordinary event [40]. This section contains an intriguing discussion of the application of ECG signal anomaly detection.

The article "Classification of Electrocardiography Hybrid Convolutional Neural Network-Long Short Term Memory with Fully Connected Layer" was published in 2022. Journal: Comput Intell Neurosci.

### 3.2. Enhanced Data

For each ailment type, incomplete data are collected due to an imbalance caused by a database that only contains the most common rhythm kinds. Data expansion can be used to generate a small amount of data in the class and reduce overfitting challenges to an acceptable level as a result of the uneven quantity of data in each data classification [41]. If the image is better, the data computation will be more efficient. Due to a loss in ECG signal training, the vast majority of earlier electrocardiogram rhythmic medications were unable to physically add information regarding expansion. In feed-forward neural networks (FFNNs) and support vector machines (SVMs), the goal of classifiers is to consider each ECG signal to have the same categorization meaning. Many studies employ the ECG signal separation approach to separate 1D ECG data into various segments in order to increase the number of data measurements while dealing with enormous volumes of information [42].  Figure 4 shows the various types of ECG signals that were obtained through the use of enhanced data (see text for explanation). Although the ECG data produced by the model in this work necessitate an image improvement strategy, the information computation should be created rather than the information enhancement technique. A 2D ECG image that has already been modified is merged with image processing to bring out the finer features. Data are collected in such a way as to focus on the ECG's image change while retaining an unaltered approximation of the outcome as a result of the data collection. By improving the exam's knowledge irregularity, this is made possible by enhancing the original functioning in a key way.

### 3.3. Fully Connected Layer [CNN-LSTM]

Deep learning is essential for both machine learning and pattern identification. Data-driven machine learning is a subset of deep learning. During this research, eight unique ECG signal patterns were identified and classified. A cross-learning approach is used to help students acquire more in-depth knowledge. The model includes all of the components, including CNN and LSTM. CNNs are better suited for geographical or private data, while LSTMs are better suited for time-series data. The LSTM layer 10 is the most commonly employed of the convolutional layers 1 through 9. Taking advantage of a completely linked layer, the process end improves its performance. Once the spatial aspect reference has been generated by using an appropriate convolutional layer, it may then be used to produce it. Such markings can be detected with the help of the LSTM layers that are created as a result of this process [43]. There is an LSTM and a CNN in the mix (none, 16, 16, 256). This is how the output looked until the model's pooling stage. The information size of an LSTM layer changes when we apply the reshape technology to reshape the model's components (256, 256). After breaking down the LSTM's temporal properties, the model is able to distinguish ECG signals across the fully linked layer. Optimizing your pattern's early stages is made easier by setting a streamlining agent and learning rate. It was in response to this that researchers created a 0.001 learning speed and a streamlining booster that are currently in use.  Figure 5 shows the proposed network mode.

The article "Classification of Electrocardiography Hybrid Convolutional Neural Network-Long Short Term Memory with Fully Connected Layer" was published in 2022. Journal: Comput Intell Neurosci.

### 3.4. Architecture and Details

The core of the proposed system, which contains the 2D CNN, is composed of three convolution blocks and a stage size of one. In addition, this is the most challenging component of the proposed design. In order to complete each convolution, an exponential linear unit is used (ELU). This layer of batch normalisation has been incorporated into the system to ensure that activation costs are consistent across batches. Each convolution is made up of two 2D CNN layers and one overall batch layer. To obtain the convolution part of a convolution task, the superposition matrix is multiplied by both of the convolution functions. It does not matter what kind of convolution is used. Pool channels with maximum step sizes of two are used for light extraction after a 2D convolution on the feature map. Compositing this feature map was difficult due to a large portion of the more intricate area being removed and labelled as a separate feature map. The groundwork for the design is being done on a daily basis. As the model structure is optimized, the feature map size is gradually decreased. This is done in order to get the most out of the model structure in terms of learning rate. Finally, each feature map is shifted to the LSTM layer in order to obtain any temporal information that is accessible. Convergence and convolution result in the highlights being broken up into numerous pieces. The LSTM circular chain method is used to predict time series. LSTM is not precisely the same as a normal RNN in terms of performance as an alternative version of a single neural network. It focuses on certain cell states and makes use of gated units to do this. Data transferred across the network must be handled consistently and efficiently, which is why LSTM regularly consolidates these systems. For modules that are part of this process, a gradient is eliminated so that long-term reliance issues can be estimated. Following an LSTM layer, a fully connected softmax system with five output neurons is used, which is controlled by a feature vector that illustrates the picture via time-dependent features. A prediction of an arrhythmia is made using the outputs of these five classifications. They are all interconnected layers.

The article "Classification of Electrocardiography Hybrid Convolutional Neural Network-Long Short Term Memory with Fully Connected Layer" was published in 2022. Journal: Comput Intell Neurosci.

As an input to the network, the layer broadcasts logical vectors on one side and vectors on the other. The facts are geared. We use a log-mel with 40 dimensions in every frame of our work. We may be able to lessen the frequency variations of the input signal by first running the signal through numerous additional convolutional layers. The architecture of each CNN layer is described, and facts are geared towards it; we employ two convolutional layers, each of which contains 256 feature maps, for a total of eight CNN layers. A recurrent 9 × 9 time channel is used for the first convolutional layer, which is followed by a 4 × 3 channel for the second convolutional layer, with the channels being distributed throughout the whole frequency range of the signal. It will be necessary to use maximum pools that are not protected in order to pool, and repetitive pooling will simply occur [44]. First, a pooling depth of three was included into the design of the first layer, and no second layer pooling was performed.

As a result of the huge number of feature maps multiplied by frequency multiplied by time, the final layer of a CNN is massive. As shown in Figure 6, such lines have their feature size reduced by a linear layer until they reach the LSTM layer. At every step of the CNN layering process, the inclusion of these linear layers has been taken into consideration, as seen in [45]. During our experiments, we noticed that reducing the size of the linear layer outputs was important to obtaining 256. In order to display the signal in real time, we send the CNN output through LSTM layers if the frequency is exhibited. We employ two LSTM layers, the first with an 832-cell LSTM layer and the second with a dimensionality reduction of 512 projection layer units, in accordance with the proposed approach. Backpropagation through time (BPTT) can only begin once the LSTM has been unrolled a total of twenty times. As a result, DNNs demonstrate how data from the hypothetical frame may be used to make a more accurate forecast of the actual frame. Each letter of the alphabet has its own unique set of LSTMs, so the data used in the CNN include a mix of letters from both alphabets. There should never be more than five possible decoding CLDLN objects in the LSTM, so that certain attributes can be preserved by setting *r* = 0. Finally, we pass the LSTM output to a pair of fully coupled DNN layers following the frequency and worldly examples. According to [46], the higher layers can provide higher specifications, which can be separated much more efficiently at each level as demonstrated in [47]. These higher specs are illustrated in [46]. 1,024 hidden units can be found in each linked layer, making up the total number.

The article "Classification of Electrocardiography Hybrid Convolutional Neural Network-Long Short Term Memory with Fully Connected Layer" was published in 2022. Journal: Comput Intell Neurosci.

The ELU study was employed in this analysis because it reveals that ECG arrhythmia was the best grouped of the conditions studied. ELU is shown in the following equation:

(1) $$\begin{array}{c} \text{RELU}\left(a\right)\;=\;\left\{\begin{array}{cc} a, & a\;\geq \;0\\ \beta \left(e^{a}-1\right), & a\;<\;0 \end{array}\right.. \end{array}$$

A mean squared error (MSE) specified in (2) shall be used to reconstruct between the input signal and output signal $\hat{a}$.

(2) $$\begin{array}{c} \text{MSE }=\;\frac{1}{N}\;\sum_{t=1}^{N}{\left(a\;-\;\hat{a}\right)}^{2}. \end{array}$$

When it comes to batch normalisation, equation (3) was computed.

(3) $$\begin{array}{c} \mu \;=\;\frac{1}{N}\;\sum_{t=1}^{N}a_{t},\\ \sigma^{2}\;=\;\frac{1}{N}\;\sum_{t=1}^{N}a_{t}\;-\;\mu ,\\ a\left(t\right)\;=\;\frac{a_{t}\;-\;\mu }{{\sqrt{\sigma^{2}\;+\varepsilon }}^{\prime }}. \end{array}$$

Overfitting is a serious problem when developing a model for training purposes. A training model is overfitted in this case, and the regularization of the dropout is employed to avoid this from happening. At the same time, we offer correlations with models in which dropout regularization could not be applied at the same level as dropout regularization. As part of the dropout regularization process, a portion of each hub in a comparable layer is likely to be eliminated in order to lessen conditions between layers. When the neurons exit, the corresponding weight will be forbidden, resulting in a significant increase in the capacity of the model. The model beyond regularization incorporates all weights into the learning process during the training period, resulting in a significant increase in the connection between the layers and the inability to perform overfitting. Dropout regularization was tested on a model with a single completely connected layer, and it was discovered to be situated at the final totally connected layer. The dropout rate had been 0.5% at the time.

The article "Classification of Electrocardiography Hybrid Convolutional Neural Network-Long Short Term Memory with Fully Connected Layer" was published in 2022. Journal: Comput Intell Neurosci.

## 4. Result and Discussion

In this study, the intention of the unbalanced classification of ECG signal was applied in the CNN-LSTM arrangement in order to get the desired results. The ECG beat data were classified according to the LSTM model, and then we used FCL to construct a CNN-LSTM configuration for classification. The acceptable practicality of a completely linked layer for the kind of ECG unbalanced rhythms was immediately apparent. We were able to establish the validity of the LSTM network topology via the use of comparison and best in class methodologies. The suggested model was mostly based on the MIT-BIH arrhythmia database, which was the primary source. Following the specifications of the AAMI standards, all MIT-BIH beats are grouped into five primary categories. This is, however, not always a desired outcome. The kind of arrhythmia will be determined by the ECG beat and the precision with which the beat shapes are formed.

The results of the PTB diagnostic ECG database were utilised to evaluate the outcomes of the MIT-BIH arrhythmia technique. A PTB reference has been created by taking 185 subjects from each of these bad issues plus 25 subjects from 12 separate meetings and merging them together (2 from PTB and 10 from MIT-BIH). As a consequence, we look at 185 examples of good and embarrassing products that can be created right now but are not because the machine is not set up to do them. F1 scores are used to describe the results of our research since we take into account and evaluate their validity.  Table 1 shows that the impacts on the standard class, including the F1 score, precision, and analysis, are both raised and broadened in every situation. As a result, the total number of ECG signals that have been labelled as normal but are actually problematic has fallen dramatically (from 16,550 to 16,575). It is clear from Table 1 that the F1 score for minorities has risen significantly. As of this writing, S has an accuracy percentage of 97.23%, while F has an accuracy rating of 96.42. Changes in other significant tactics employed in authoring quality networks are shown in Table 2. Using a dropout regularizer, we predicted that the latent vector would show more prominently while remaining as flat and stable as possible. Money is required to restructure the input signal in more significant ways. The data we have gathered show that regularization frequently enhances the model and generally improves the model's accuracy, as we have shown.  Table 3 shows the experimental results of the MIT-BIH dataset model.

Figure 6 depicts the accuracy and loss as a result of modifications to the training and test conditions. To ensure a steady condition throughout the training, the model was verified after about 35 epochs of training in this mode of operation. In order to estimate the model's deal performance, the following performance metrics were used: accuracy, R-squared, root mean square error, and computation time. After exploratory testing, the CNN-LSTM combined with the FCL hybrid model achieved 99.43% accuracy, 0.884% R-squared, 0.18% RMSE, and a 20% reduction in calculation time, among other results.  Figure 7 depicts the many forms of heart illnesses that have been categorized according to the suggested design. We may deduce the five forms of sickness from this chart, and we can also look at the length of the R-R gap between the peak and the valley.

The article "Classification of Electrocardiography Hybrid Convolutional Neural Network-Long Short Term Memory with Fully Connected Layer" was published in 2022. Journal: Comput Intell Neurosci.

Table 2 shows that our suggested CNN-LSTM and FCL algorithms perform exceptionally well. As in earlier investigations, we used deep learning to establish how ECG irregular beat information was to be categorized in the classification process. We used LSTM with FCL to classify ECG arrhythmias that were out of balance. The categorization of imbalanced ECG data is frequently employed, according to studies [21, 43]. When it comes to the most important difference, we employ FCL to adjust the loss function in order to focus on ECG beats that appear to be misclassified, hence increasing the accuracy of arrhythmia classification. In terms of recall, our CNN-LSTM with FCL achieves the highest results on the dataset. As a result, inappropriate results, such as aberrant ECG beats, are incorrectly ascribed to regular ECG beats, according to this hypothesis.

## 5. Conclusions

The initial analysis of cardiovascular infection is based on the study and differentiation of arrhythmic indications and symptoms. CNN-LSTM and FCL interplay was recommended in this study to enhance readiness while limiting the impact of an immense amount fundamental specific ECG beat information on the model training. However, the proposed architecture uses LSTM layers to move the variation to the outputs of DNN layers that have large effective feature illustration than the CNN layers, which diminish every spectral fluctuation in the input feature. For CNN-LSTM and FCL, the results show that they achieved 99.43% accuracies (F1 score), 96.27% precision (precision), 94.85% recall (recall), and 92.85% precision (precision). According to the results of the MIT-BIH arrhythmic test, the proposed design was appropriate and had a high intensity level. Cardiologists could use the method outlined here to help them make more accurate and unbiased diagnoses of ECGs in telemedicine situations. Finally, future evaluations will include additional types and beats with various degrees of difficulty. In addition, we propose to present exact rates of noise to ECG data in order to research the presence of CNN-LSTM by means of FCL pattern in order to investigate its appearance.

The article "Classification of Electrocardiography Hybrid Convolutional Neural Network-Long Short Term Memory with Fully Connected Layer" was published in 2022. Journal: Comput Intell Neurosci.

## Figures and Tables

**Figure 1:** Normal ECG sinus rhythm.

**Figure 2:** Proposed framework for ECG arrhythmia classification.

**Figure 3:** ECG data preprocessing.

**Figure 4:** Enhanced data in one heartbeat of each category.

**Figure 5:** Flow diagram of fully connected layer - CNN-LSTM.

**Figure 6:** Block diagram of CNN-LSTM with fully connected layer.

**Figure 7:** Classification of different heart diseases.

**Table 1:** Experimental results of the architecture performance.

Parameter	CNN-LSTM	CNN
R-squared	0.884	0.826
Accuracy	99.43%	98.61%
MAE	0.027	0.020
RMSE	0.18	0.08
Training time (s)	235.34	255.62

**Table 2:** Comparison of proposed method with existing methods.

Authors	Approach	Year	Num. of classes	Accuracy (%)	F1 score	Precision	Recall
[9]	Wavelet + BiLSTM	2018	5	99.25	—	—	—
[10]	NB, SVM, MLP, and OPF	2019	5	94.30	—	—	—
[21]	CAE and LSTM	2019	5	99.00	—	—	99.00%
[23]	Deep residual network	2020	5	99.06	—	96.76	93.21%
[35]	LSTM	2020	5	99.37	95.77%	96.73%	94.89%
[43]	CNN-LSTM	2020	8	99.01	—	—	—
Proposed method	Fully connected CNN-LSTM	2022	5	99.43	96.27%	94.85%	92.85%

**Table 3:** Experimental results of the MIT-BIH dataset model.

Class	CNN-LSTM			CNN		
	F1 score	Precision	Recall	F1 score	Precision	Recall
V	94.23	99.31	90.14	92.41	94.34	91.76
S	97.23	100	83.26	82.19	86.46	77.52
N	94.32	82.53	99.17	99.17	98.74	98.93
Q	99.14	98.89	98.43	96.15	98.18	97.81
F	96.42	93.51	93.26	83.57	82.98	79.27
Average	96.27	94.85	92.85	90.69	92.14	89.06

## Data Availability

The data used to support the findings of this study are available from the corresponding author upon reasonable request.
